The article "Leukocyte telomere length and obesity in children and adolescents: A systematic review and meta-analysis" was retracted in 2023. Reason: concerns about the authorship.

# Leukocyte telomere length and obesity in children and adolescents: A systematic review and meta-analysis

**DOI:** 10.3389/fgene.2022.861101

**Published:** 2022-09-07

**Authors:** Mohammad Saeed Kahrizi, Indrajit Patra, Abduladheem Turki Jalil, Harun Achmad, Samira Alesaeidi, Moaed E. Al-Gazally, Sogol Alesaeidi

**Affiliations:** ^1^ Department of Surgery, Alborz University of Medical Sciences, Karaj, Alborz, Iran; ^2^ An Independent Researcher, PhD from NIT Durgapur, Durgapur, West Bengal, India; ^3^ Medical Laboratories Techniques Department, Al-Mustaqbal University College, Babylon, Iraq; ^4^ Department of Pediatric Dentistry, Faculty of Dentistry, Hasanuddin University, Makassar, Indonesia; ^5^ Department of Internal Medicine and Rheumatology, Rheumatology Research Center, Tehran University of Medical Sciences, Tehran, Iran; ^6^ College of Medicine, University of Al-Ameed, Karbala, Iraq; ^7^ Department of Pediatric Medicine, Imam Hossein Hospital, Isfahan University of Medical Sciences, Isfahan, Iran

**Keywords:** leukocyte telomere length, obesity, LTL, children, adolescents, youth

## Abstract

**Background:** Several studies have revealed the negative effects of adiposity on telomere length shortening. However, the results of the studies assessing the negative relationship between obesity and leukocyte telomere length (LTL) are not consistent. This systematic review and meta-analysis are aimed to pool the results of articles assessing the relationship between obesity and LTL among children and adolescents.

**Methods:** To retrieve the related studies, four online databases including PubMed, Embase, ProQuest, and Scopus were searched until May 2022. Observational studies evaluating the relationship between obesity and LTL among apparently healthy children and adolescents (aged ≤18 years) were included in the study. We considered the studies that had reported a mean ± standard deviation of LTL. The random-effects model was used to assess the pooled weighted mean difference (WMD) and a 95% confidence interval (CI).

**Results:** The search yielded seven studies from an initial 3,403 records identified. According to the results of seven articles with 4,546 participants, obesity was associated with LTL shortening among children and adolescents (WMD = −0.081; 95% CI: −0.137 to −0.026; *p* = 0.004; I^2^ = 99.9%). Also, no publication bias was observed. According to the results of subgrouping, significant results were only attributed to the studies conducted in Europe, with high quality scores, among overweight and obese adolescents, with a baseline LTL lower than 1, and performed in community-based school settings. Also, according to the subgrouping and meta-regression results, the obesity definition criteria and baseline LTL were the possible sources of between-study heterogeneity.

The article "Leukocyte telomere length and obesity in children and adolescents: A systematic review and meta-analysis" was retracted in 2023. Reason: concerns about the authorship.

**Conclusion**: We observed shorter LTL among overweight and obese children and adolescents. To obtain more reliable results, further longitudinal prospective studies with large sample sizes and more consistent and accurate definitions of obesity are required.

## Introduction

Telomeres are non-coding repeated sequences of genome that are responsible in maintaining DNA integrity and stability during each division (Flannagan et al., 2020; Tang et al., 2020). With each cell division, the telomere length shortens and this shortening does not occur at a constant rate, but rather, rapidly declines from birth through age 4 (Rufer et al., 1999; Gasmi et al., 2021). The normal telomere length of an adult human is approximately 10–15 thousand base pairs (bp), while the protruding part of the G-chain, including 150–200 bp, can bend and form a loop structure (T-loop) (Zimnitskaya et al., 2022), telomeres shorten ~100 bp for each cell division as a result of incomplete replication and exposure to oxidative stress and inflammation (Wojcicki et al., 2016a).

Leukocyte telomere length (LTL) in early childhood is a predictor of its size in adulthood (Dalgård et al., 2015). Numerous genetic and environmental factors might affect LTL among children and adolescents. Several studies revealed that dietary ingredients, including maternal folate (Entringer et al., 2015), blood vitamin D concentrations (Kim et al., 2017), dietary zinc status (Milne et al., 2015), and dietary antioxidant status (García-Calzón et al., 2015) could affect LTL in newborns. Moreover, some other environmental factors might affect LTL, among which the role of obesity in shortening LTL is of great importance (Strandberg et al., 2011; Chen et al., 2014; Mazidi et al., 2018; Rojas et al., 2018; Zgheib et al., 2018; Aghajani et al., 2020). A recent meta-analysis of cross-sectional studies showed a converse association between body mass index (BMI) and relative LTL in adults (Gielen et al., 2018). Results from two studies showed that an increase in adiposity measures was related to a decrease in LTL (Rehkopf et al., 2016; Batsis et al., 2018). The observed association between LTL and obesity might also be described by the obesity-associated (FTO) gene-involved pathways and fat mass (FM) (Zhou et al., 2017; Colon et al., 2019). Shorter telomeres have been related to increasing BMI and more recently with increasing waist circumference (WC) and waist-to-hip ratio (WHR) in women (Nordfjäll et al., 2008). A higher WHR is considered an independent predictor of TL shortening, and abdominal obesity seems to have a robust influence on telomere shortening (Farzaneh-Far et al., 2010).

The article "Leukocyte telomere length and obesity in children and adolescents: A systematic review and meta-analysis" was retracted in 2023. Reason: concerns about the authorship.

According to Brandao CFC et al. (Brandao et al., 2020), central obesity might affect the telomere structure that could be modified by physical training. In a study conducted on 145 healthy infants, LTL shortening from 3 months to 2 years related to FM %, visceral FM, and FM index at 2 years of age, and LTL shortening tended to associate with the gain in FM % from three to 6 months (de Fluiter et al., 2021). Lee M et al. (Lee et al., 2011) reported that visceral adipose tissue, BMI, and total body fat were related to a shorter telomere length. Previous studies investigating the role of childhood obesity in LTL shortening have inconsistent results. In a study by Clemente DBP et al*.*, 1,396 mother–child pairs of the multi-center European birth cohort study (HELIX), higher childhood adiposity markers such as FM, skinfold thickness, WC, and BMI were associated with a shorter LTL among eight-year-old children (Clemente et al., 2019). In another study by Buxton JL et al. (Buxton et al., 2011), LTL was shorter among 793 obese French children aged 2–17 years old compared to non-obese children. However, several other studies did not report a significant association between obesity markers and LTL among children and adolescents (Theall et al., 2019; Flannagan et al., 2020; Todendi et al., 2020).

Childhood obesity is a global epidemic and a predictor of obesity and associated co-morbidities, including cardiovascular events, diabetes, and several types of cancers in adulthood (Bridger, 2009; Schroeder et al., 2020; Zhou et al., 2021; Nasiri, 2022). On the other hand, a shorter LTL is a predictor of numerous diseases such as myocardial infarction (Bekaert et al., 2007; Koriath et al., 2018), type 2 diabetes (Tamura et al., 2016; Wang et al., 2016), non-alcoholic fatty liver disease (Kar and Khandelwal, 2015; Zhang et al., 2019a; Jabbar, 2022), stroke (Emami et al., 2019; Tian et al., 2019; Al-Obaidi et al., 2022), glucose intolerance (Grunnet et al., 2019; Weale et al., 2019), and a higher all-cause mortality among adults (Fitzpatrick et al., 2011; Strandberg et al., 2011; Mons et al., 2017).

In a recent systematic review and meta-analysis by Lin L et al. (Lin et al., 2021), a lower LTL was reported in obese children compared to non-obese ones (SMD: −0.85; 95% CI: −1.42 to −0.28; *p* < 0.01). However, they reported the results by fixed effects model, in which the major assumption is that the true effect is the same in all studies. This assumption may be implausible in many systematic reviews because the expectation is that the effect size is similar but not identical across studies, and this between-study variability is considered only in the random effects model (Borenstein et al., 2007; Naghibi et al., 2021). Also, two other meta-analyses reported an inverse association between LTL and general and central obesity among adults (Abolhasani-Zadeh et al., 2021; Abbasalizad Farhangi and Nikniaz, 2022).

The article "Leukocyte telomere length and obesity in children and adolescents: A systematic review and meta-analysis" was retracted in 2023. Reason: concerns about the authorship.

In a meta-analysis conducted by Lin L et al., not all the eligible studies were included possibly due to the time of publication (Zhu et al., 2014; Flannagan et al., 2020), and the LTL unit in all the included studies was not identical. For example, they included the study by Buxton L et al. in the meta-analysis and reported the log T/S ratio and not the unchanged variable. They also included the study by Zannolli R et al. (Zannolli et al., 2008) that measured the LTL by terminal restriction fragments (TRF) and not the T/S ratio. Considering such discrepancies and because of the importance of the association between LTL and childhood obesity, this systematic review and meta-analysis evaluated the published cross-sectional studies to assess the relationship between obesity and LTL among children and adolescents.

## Methods and materials

We used Preferred Reporting Items for Systematic Reviews and Meta‐Analyses (PRISMA) for reporting the results (Supplementary Table S1) (Moher et al., 2009).

### Search strategy

In this study, four electronic databases, including PubMed, Embase, ProQuest, and Scopus were systematically searched. A total of 3,403 articles evaluating the association between obesity and telomere length among children and adolescents were retrieved up to May 2022. No language restriction was applied. We also performed a hand-search from all other available documents, reference lists of all articles, and gray material to find any possible missed publications. The search strategy was created with a combination of the MeSH (Medical Subject Headings) terms from the PubMed database and free text words. A sample search strategy for PubMed is presented in Supplementary Table S1.

### Selection of the studies

Our search strategy resulted in the retrieval of a total of 3,403 articles. After removing the duplicates, 2,299 articles remained. Three independent investigators checked the remaining articles. Next, 1,223 articles were excluded after screening the titles and abstracts. Out of 1,076 remaining articles, 1,069 articles were excluded due to irrelevant designs, subjects, other age groups, conferences, congresses, and seminars. Some of the excluded studies did not evaluate the requested association of the studied parameters. Any discrepancies between reviewers were resolved by discussion. Consequently, seven articles were included in the final meta-synthesis (Figure 1). The PICO model (patients, intervention, comparison, and outcome), as one of the most widely used models for formulating clinical questions, was used for selecting the studies in the meta-analysis (Table 1).

The article "Leukocyte telomere length and obesity in children and adolescents: A systematic review and meta-analysis" was retracted in 2023. Reason: concerns about the authorship.

**FIGURE 1:** Study flowchart.

**TABLE 1:** The PICO criteria used for the systematic review.

PICO criteria	Description
Participants	Children and adolescent population
Exposure (Interventions)	Children with overweight or obesity
Comparisons	Children without overweight or obesity
Outcome	Leukocyte telomere length as T/S ratio
Study design	Observational studies with the design of cross-sectional, case control or cohort studies with the baseline data of requested variables

### Inclusion and exclusion criteria

The inclusion criteria were as follows: 1) Cross-sectional studies; 2) studies evaluating the relationship between LTL and obesity measurements such as BMI; 3) studies conducted among children and adolescents (aged ≤18 years); 4) studies providing the odds ratio of the association between LTL and obesity measurements; 5) studies providing the mean ± standard deviation (SD) of LTL among the youth with or without obesity; and 6) studies recruiting only healthy young people.

### Data extraction and risk of bias assessment

The name of the first author, journal name, year of publication, region, age range of participants, study design, total number of participants, setting, adjusted covariate, gender, LTL measurement tools, and main findings were collected. The Agency for Healthcare Research and Quality (AHRQ) checklist was used for the risk of bias assessment (Cho et al., 2017) (Table 2).

**TABLE 2:** Risk of bias assessment using the Agency for Healthcare Research and Quality (AHRQ) checklist.

ARHQ methodology checklist items for cross-sectional study	Todendi PF (Todendi et al., 2020)	Flannagan KS (Flannagan et al., 2020)	Theall KP (Theall et al., 2019)	Lamprokostopoulou a (Lamprokostopoulou et al., 2019)	Wojcicki JM (Wojcicki et al., 2016a)	Zhu H (Zhu et al., 2014)	Al-Attas OS (Al-Attas et al., 2010)
1) Define the source of information (survey, record review)	⊕	⊕	⊕	⊕	⊕	⊕	⊕
2) List the inclusion and exclusion criteria for exposed and unexposed subjects (cases and controls) or refer to previous publications	⊕	U	⊕	⊕	⊕	⊕	⊕
3) Indicate the time period used for identifying patients	⊕	⊕	⊕	⊕	⊕	⊕	⊕
4) Indicate whether or not subjects were consecutive if not population-based	⊕	⊕	⊕	⊕	⊕	⊕	⊕
5) Indicate if evaluators of subjective components of study were masked to other aspects of the status of the participants	U	U	U	U	U	⊕	U
6) Describe any assessments undertaken for quality assurance purposes (e.g., test/retest of primary outcome measurements)	⊕	U	U	U	U	U	U
7) Explain any patient exclusions from analysis		⊕	⊕	⊕	⊕	⊕	U
8) Describe how confounding was assessed and/or controlled	⊕	⊕	⊕	⊕	⊕	⊕	⊕
9) If applicable, explain how missing data were handled in the analysis	U	U	⊕	U	⊕	U	⊕
10) Summarize patient response rates and completeness of data collection	U	U	⊕	⊕	⊕	U	U
11) Clarify what follow-up, if any, was expected and the percentage of patients for which incomplete data or follow-up was obtained	⊕	U	U	U	U	U	U
Final score	7	5	8	7	8	7	6

L, low risk of bias; H, high risk of bias; U, unclear risk of bias. The items were scored as follows: if the answer were “YES,” the score was “1” and if the answers were “NO” or “UNCLEAR”, the score was “0”. The final quality scores were: low quality = 0–3; moderate quality = 4–7 and high quality ≥8. ⊕, presence of the criteria, U, unclear.

The article "Leukocyte telomere length and obesity in children and adolescents: A systematic review and meta-analysis" was retracted in 2023. Reason: concerns about the authorship.

### Statistical analysis

Data analysis was performed by STATA version 13 (STATA Corp, College Station, TX, United States). *p*-values less than 0.05 were considered as statistically significant. No study evaluated the odds ratio (OR) of the association between obesity and LTL among children and adolescents. Therefore, two meta-analyses that reported the comparison of the relative telomere length [mean ± SD] in obese versus non-obese children and adolescents were included. The mean and SD of LTL were used to calculate the unstandardized effect size calculated by the pooled estimate of weighted mean difference (WMD) with a 95% confidence interval (CI). A meta-regression fitting was done for several variables, including weight status, continent, baseline telomere, quality score, sample size, age, gender, and setting for identifying the source of heterogeneity. Between-study heterogeneity was performed by Cochran’s Q and I^2^ tests (Higgins and Thompson, 2002). For significant heterogeneities of either the Q statistic with *p* < 0.1 or I_2_ >50%, the random effects model was used (Riley et al., 2011). Also, we used the random effects model because between-study heterogeneity is considered only in this model. Subgrouping was also performed to identify the source of heterogeneity. Begg’s funnel plots followed by Begg’s adjusted rank correlation and Egger’s regression asymmetry tests were used to assess publication bias.

### Definitions and measurements

In the current meta-analysis, as previously described by the World Health Organization (WHO), a child was defined as aged under 10 years and an adolescent as aged between 10–19 years (Organization, 2020). In all the included studies, the mean LTL measurement was determined from leukocyte DNA by a modified quantitative polymerase chain reaction (PCR)-based method, as previously described (Cawthon, 2002; Zhu et al., 2014). The relative ratio of the telomere repeat copy number (T) to a single copy gene copy number (S) was determined by PCR and the T/S ratio was calculated for each individual. As described in Table 3, the obesity criteria were based on three standard definitions. First, based on the WHO definition of BMI Z-score ≤ +1 SD as normal weight; > +1SD as overweight; and > +2SD as obese (Onis et al., 2007); second, based on the International Obesity Task Force (IOTF) cut‐off points of BMI of 18.5–24.9 and ≥30 kg/m^2^ as overweight and obese, respectively (Cole and Lobstein, 2012); and third, based on the Centres for Disease Control and Prevention’s (CDC) growth charts (Kuczmarski, 2000), sex-specific BMI-for-age at or above the 85th percentile but less than the 95th and ≥95th percentile were defined as overweight and obese, respectively.

The article "Leukocyte telomere length and obesity in children and adolescents: A systematic review and meta-analysis" was retracted in 2023. Reason: concerns about the authorship.

**TABLE 3:** Characteristics of the studies included in the meta-analysis owing to report the comparison of telomere length among obese and non-obese children and adolescence.

First author/year	Journal/Country	Setting	Study population/Num	Age range (y)	Male %	Overweight/obesity status	Obesity criteria	Main finding
Todendi PF (Todendi et al., 2020)/2020	Nutrition/Brazil	School	Healthy/981	7–17	44.03	Overweight/obesity with 42% overweight	BMI for age Z score > +1SD, overweight; and >+2 SD obesity	No significant difference in telomere length between obese and non-obese children and adolescence
Flannagan KS (Flannagan et al., 2020)/2020	Eur J Nut/Colombia	School	Healthy/723	5–12	45.6	Overweight/obesity	BMI for age Z score > +1SD, overweight; and >+2 SD obesity	Non- significant decrease and increase in telomere length with increased BMI among girls and boys respectively
Theall KP (Theall et al., 2019)/2019	Prev Med Rep/United States	Community	Healthy/90	5–16	46	Overweight/obesity with 32% overweight	≥85th and ≥95th percentile of BMI for overweight and obesity respectively	Non-significant decrease in telomere length among obese pediatric
Lamprokostopoulou A et al. (Lamprokostopoulou et al., 2019)/2019	Eur J Clin Invest/Greece	School	Healthy/919	9–13	50.27	Overweight/obesity with 30.03% overweight	BMI:25–29.9 and ≥30 kg/m^2^ for overweight and obesity respectively	Significantly lower telomere length in overweight and obese compared with non-obese children (*p* = 0.002)
Wojcicki JM (Wojcicki et al., 2016a)/2016	Am J Clin Nutr/United States	Community	Healthy/400	4–5	46.8	Obesity	≥85th and ≥95th percentile of BMI for overweight and obesity respectively	Non-significant shorter telomere length in obese versus non-obese children
Zhu H (Zhu et al., 2014)/2014	Int J Obese/Georgia	Community	Healthy/766	14–18	50	Overweight/obesity	≥85th and ≥95th percentile of BMI for overweight and obesity respectively	Non-significant shorter telomere length in obese versus non-obese adolescents
Al-Attas OS (Al-Attas et al., 2010)/2010	Acta Pædiatrica/Saudi Arabia	Community	Healthy/148	5–12	46.6	Obesity	BMI:25–29.9 and ≥30 kg/m^2^ for overweight and obesity respectively	Significantly lower LTL among obese boys (*p* = 0.049); but no significant difference among girls

The study by Todendi PF et al. (Todendi et al., 2020) was performed in children and adolescence separately so the results were included as two independent studies. The studies by Flannagan KS et al (Flannagan et al., 2020) and Al-Attas OS (Al-Attas et al., 2010) were included as two independent studies among boys and girls. The study by Lamprokostopoulou A et al. (Wojcicki et al., 2016b) was included as two independent studies in overweight and obese individuals. The study by Wojcicki JM et al. (Wojcicki et al., 2016a), was performed in two different age groups of 4 and 5 years old, thus, the results were included as two independent studies. All of the studies were conducted in combination of both genders and had cross-sectional design. LTL assessment was based on modified quantitative polymerase chain reaction polymorphism q (PCR) and was expressed as relative ratio of telomere repeat copy number (T) to single copy gene copy number (S) or T/S ratio.

The article "Leukocyte telomere length and obesity in children and adolescents: A systematic review and meta-analysis" was retracted in 2023. Reason: concerns about the authorship.

## Results

### Study characteristics

The characteristics of the included studies are presented in Table 3. Totally, seven articles reporting the LTL among children and adolescents with or without obesity were evaluated. However, some studies had more than one individual report. For example, the study by Todendi PF (Todendi et al., 2020) had been performed separately among children and adolescents; so, the results were included as two independent studies. Similarly, the studies by Flannagan KS et al. (Flannagan et al., 2020) and Al-Attas OS (Al-Attas et al., 2010) were included as two independent studies among boys and girls and the study by Lamprokostopoulou A et al. (Wojcicki et al., 2016b) was included as two independent studies in individuals with obesity. Also, the study by Wojcicki JM et al*.* had been performed in two different age groups of four- and five-year-old children; thus, the results were included as two independent studies. Moreover, they used dried blood spots to measure LTL by qPCR (Wojcicki et al., 2016a). Therefore, 12 individual reports with a total of 4,546 participants were included in the meta-analysis. All the included studies had a cross-sectional design, they had been performed among healthy youth, and the relative telomere length assay method was qPCR. Six studies extracted genomic DNA using whole blood samples, and one study used dried blood spots (Wojcicki et al., 2016c). All the included studies measured the telomere length from leukocytes. Three studies (Lamprokostopoulou et al., 2019; Flannagan et al., 2020; Todendi et al., 2020) had been performed in a school setting and four studies (Al-Attas et al., 2010; Zhu et al., 2014; Wojcicki et al., 2016a; Theall et al., 2019) were community-based. Four studies (Al-Attas et al., 2010; Zhu et al., 2014; Wojcicki et al., 2016a; Lamprokostopoulou et al., 2019) included only youth with obesity, while three studies (Theall et al., 2019; Flannagan et al., 2020; Todendi et al., 2020) included children and adolescents with obesity. Two studies (Wojcicki et al., 2016a; Theall et al., 2019) had been performed in the United States, one in Brazil (Todendi et al., 2020), one in Greece (Lamprokostopoulou et al., 2019), one in Colombia (Flannagan et al., 2020), one in Georgia (Zhu et al., 2014), and one in Saudi Arabia (Al-Attas et al., 2010). The study by Wojcicki JM et al*.* (Wojcicki et al., 2016a) had been performed only among children and the study by Lamprokostopoulou A et al*.* (Lamprokostopoulou et al., 2019) included only adolescents; other studies involved both children and adolescents. The studies by Lamprokostopoulou A et al. (Lamprokostopoulou et al., 2019) and Al-Attas OS et al. (Al-Attas et al., 2010) reported a significantly lower LTL among overweight and obese youth compared to non-overweight and non-obese ones. While four studies (Zhu et al., 2014; Wojcicki et al., 2016a; Theall et al., 2019; Flannagan et al., 2020) reported a non-significantly lower LTL among overweight and obese youth, one study reported no difference (Todendi et al., 2020). In addition, one study that reported the average telomere length among children with type 1 diabetes was excluded from the study (Tesovnik et al., 2015).

The article "Leukocyte telomere length and obesity in children and adolescents: A systematic review and meta-analysis" was retracted in 2023. Reason: concerns about the authorship.

### The results of meta-analysis

The results of the two-class meta-analysis for the association between obesity and LTL are presented in Figure 2. The results showed that overweight and obesity were associated with a reduced LTL measured as the T/S ratio (WMD = −0.081; 95% CI: −0.137, −0.026; *p* = 0.004; I^2^ = 99.9%). To find the source of heterogeneity, subgrouping was performed for the comparison of LTL between overweight and obese youth versus non-overweight and non-obese ones (Table 4). In the subgroupings, the obesity criteria reduced the heterogeneity for obesity classification based on the WHO criteria of BMI-for-age Z score that had 0% heterogeneity. The results of meta-regression also showed the baseline telomere length and obesity criteria as possible sources of heterogeneity (reduced Tau^2^ from 0.0509 to −0.1221 and −0.131, respectively); however, this reduction was only statistically significant for the obesity criteria (Table 5). The results of the quality assessment according to the AHRQ checklist (Table 2) revealed that the quality score of all the studies was moderate or high, and there was no study with poor quality. Among the included studies, five studies had moderate quality scores and two studies had high quality scores. According to the results of Begg’s and Egger’s regression tests, no publication bias was observed (P-Begg = 0.583; P-Egger = 0.261; Figure 3).

**FIGURE 2:** Weighted mean difference (WMD) with a 95% confidence interval (CI) of the comparison of leukocyte telomere length (LTL) in children and adolescents with or without overweight/obesity.

**TABLE 4:** Results of subgroup analyses of the comparison of leukocyte telomere length (LTL) in overweight/obese versus non-overweight/obese youth.

Group	No. of studies	WMD (95%CI)	P	P _heterogeneity_	I^2^, %	P _between study heterogeneity_
Total^a^	12	−0.081 −0.137 −0.026	0.004	<0.001	99.9	
Weight status						<0.001
Overweight + Obese	8	−0.075 −0.254 0.104	0.049	<0.001	96.6	
Obese	4	−0.061 −0.151 0.030	0.087	<0.001	99.3	
Continent						<0.001
United States	8	−0.052 −0.119 0.014	0.124	<0.001	98.7	
Europe	2	−0.185 −0.214 −0.156	<0.001	<0.001	99.8	
Asia	2	−0.084 −0.310 0.141	0.463	<0.001	99.5	
Baseline LTL (T/S ratio)						<0.001
≤1	6	−0.131 −0.200 −0.062	<0.001	<0.001	100	
>1	6	−0.035 −0.090 0.020	0.216	<0.001	97.5	
Sample size						<0.001
≤100	3	−0.156 −0.391 0.078	0.192	<0.001	99.8	
100–400	5	−0.008 −0.019 0.004	0.199	0.871	-	
>400	4	−0.099 −0.180 −0.017	0.018	<0.001	100	
Quality score						<0.001
5–6	4	−0.045 −0.197 0.107	0.564	<0.001	98.4	
7–9	8	−0.098 −0.158 −0.038	0.001	<0.001	100	
Gender						<0.001
Both	8	−0.098 −0.158 −0.038	0.001	<0.001	100	
Boys	2	−0.091 −0.316 0.134	0.427	<0.001	93.6	
Girls	2	0.029 0.014 0.044	<0.001	0.311	2.5	
Age range						<0.001
Children	2	−0.007 −0.019 0.004	0.214	0.707	0	
Adolescents	1	−0.010 −0.013 −0.007	<0.001	-	-	
Children + adolescents	9	−0.121 −0.161 −0.082	<0.001	<0.001	99.8	
Setting						<0.001
School	7	−0.072 −0.139 −0.005	0.035	<0.001	100	
Community	5	−0.097 −0.200 0.006	0.065	<0.001	99.5	
Obesity criteria						<0.001
BMI-Z score for age	4	−0.006 −0.054 0.042	0.808	0.766	0	
BMI percentile	4	−0.081 −0.171 0.008	0.075	<0.001	99.5	
BMI	4	−0.184 −0.214 −0.155	<0.001	<0.001	99.5	

a Note that because all of included studies had cross-sectional designs and telomere length was assessed by qPCR, thus, subgrouping according to these parameters were not performed. Also, note that the study by Todendi PF (Todendi et al., 2020) was performed in children and adolescence; the studies by Flannagan KS et al. (Flannagan et al., 2020) and Al-Attas OS (Al-Attas et al., 2010) were performed separately in boys and girls; The study by Lamprokostopoulou A et al. (Wojcicki et al., 2016b) was performed seperaely among overweight.

The article "Leukocyte telomere length and obesity in children and adolescents: A systematic review and meta-analysis" was retracted in 2023. Reason: concerns about the authorship.

**TABLE 5:** Meta regression approach in the two-class meta-analysis.

Hypertension (HTN)	Tau^2^	*p*	95% CI
Estimate of between-study variance	0.0509		
By weight status (obese or not)	0.0602	0.39	(−0.08, 0.20)
By continent (United States or not)	0.0415	0.57	(−0.11, 0.20)
By baseline telomere as T/S ratio (>1 or not)	−0.1221	0.06	(−0.25, 0.08)
By sample size (>400 or not)	−0.0365	0.62	(−0.19, 0.12)
By quality score (>7 or not)	−0.0865	0.27	(−0.25, 0.07)
By gender (both or not)	−0.0865	0.28	(−0.25, 0.07)
By age (0–18 years or not)	−0.1094	0.10	(−0.24, 0.02)
By setting (school or not)	0.0159	0.83	(−0.14, 0.17)
By Obesity criteria (BMI-for age Z score)	−0.131	**0.049**	(−0.25, -0.10)

Statistically significant and less than 0.05 *p*-values are in bold.

**FIGURE 3:** Begg’s funnel plot [(with pseudo 95% confidence intervals (CIs)] of the weighted mean difference (WMD) versus the standard error (se) of WMD for the comparison of LTL in children and adolescents with or without overweight/obesity (P begg = 0.583; P egger = *p* = 0.261).

## Discussion

In this meta-analysis, for the first time, we identified the role of obesity in shortening LTL among apparently healthy children and adolescents. Almost all the previous meta-analyses had been performed mostly among adults (Wang et al., 2016; Gielen et al., 2018). In this meta-analysis, we summarized the results of seven articles with 4,546 participants. We also performed a subgroup meta-analysis according to weight status, continent, age range, sample size, gender, baseline telomere length, quality score, and setting. We witnessed that the effects of obesity on LTL varied according to the following parameters: studies performed in Europe, community-based studies, conducted in school settings, performed in overweight youth, having a baseline LTL (T/S ratio) less than 1, having high quality, and the existence of a significant difference between LTL in youth with or without overweight and obesity.

In a previous meta-analysis, similar to our results, a negative association was reported between LTL and BMI among adults (Gielen et al., 2018). The telomere length varied between different cell types in different subpopulations, which might explain the observed significant results among European studies (Freedman et al., 1997). Two European studies had been performed in Greece and Georgia with a mostly white population. Similarly, previous studies demonstrated that the negative effects of obesity on LTL are more pronounced among white populations (Gielen et al., 2018). Generally, the baseline LTL among white populations is lower compared to black populations due to a host of interacting biological factors, including replication rates of hematopoietic stem cells (Hunt et al., 2008). Another observation of a more pronounced reduction in LTL among those with a lower baseline LTL also confirms this finding. Hansen ME et al*.* (Hansen et al., 2016) suggested that the differences in LTL between Africans and Europeans are influenced by polygenic adaptation, and these differences might clarify, in part, the ethnic differences in risks for human diseases related to LTL. Also, population-based studies with more than 400 participants showed significant differences among LTL of youth with or without overweight and obesity. This finding highlights the effects of a large sample size in cross-sectional studies on the validity of findings. Several studies showed that in humans, a shorter adult LTL seems to be related to a suite of differences in behavior, including inactivity, obesity, smoking, alcohol intake, and higher stress reactivity (Cherkas et al., 2008; Costa et al., 2015; Mundstock et al., 2015; Müezzinler et al., 2016; Astuti et al., 2017). Although some of these relations are based on single studies and may not be vigorous, physical activity, BMI, and smoking are based on the meta-analyses of many published studies (Ulaganathan et al., 2018; Fairman et al., 2021; Kamolthip et al., 2021; Leman et al., 2021). Also, several studies revealed the possible role of environmental pollutants like air and traffic pollutants on LTL shortening; in a systematic review of more than 12,058 subjects, Zhao B et al. revealed that air pollution reduced LTL (Zhao et al., 2018), other studies also reported similar results about air pollution (Lee et al., 2019; Niehoff et al., 2019) and this finding was also confirmed in several other studies about the role of traffic pollutants (Hoxha et al., 2009), low to moderate exposure to lead (Pawlas et al., 2015). In the National Health and Nutrition Examination Survey, 1999–2002, the highest quartiles of blood and urine cadmium levels were associated with −5.54% (95% CI: −8.70, −2.37) and −4.50% (95% CI: −8.79, −0.20) shorter LTLs among 6,796 and 2,093 adults (Zota et al., 2015). Several other chemicals like phthalates and phenols are also known to affect LTL (Scinicariello et al., 2016; Zhang et al., 2022). On the other hand, several studies revealed the possible role of these pollutants and toxins in obesity development; in the study by Vafeiadi M et al. (Vafeiadi et al., 2018), early childhood exposure with phthalates was associated with obesity development in later life. Similar findings were also reported about the role of phenols, pesticides (Zhang et al., 2019b), bisphenol A (Stojanoska et al., 2017), and air pollutants (An et al., 2018) in the development of obesity. These findings highlight the mediatory role of these environmental pollutants, chemicals, and toxins in the obesity– LTL relationship among children.

The article "Leukocyte telomere length and obesity in children and adolescents: A systematic review and meta-analysis" was retracted in 2023. Reason: concerns about the authorship.

This two-class meta-analysis compared telomere length among overweight and obese children with non-overweight and non-obese ones. This is a direct, more accurate, and robust represent of the study’ parameters compared to a previous meta-analysis by Gielen M et al. (Gielen et al., 2018) on standardized regression coefficients regarding the association between BMI and telomere length in adults. The meta-analysis of the regression coefficient is a controversial issue since it belongs to the regression models that include different sets of covariates; so, it cannot be an accurate representative of the same parameter and their direct combination is meaningless (Fernández-Castilla et al., 2019).

In this meta-analysis, the obesity criteria and baseline LTL were identified as possible heterogeneity sources, even though this was just significant for the obesity criteria. In subgrouping, the heterogeneity for the WHO criteria of obesity according to the BMI-for-age Z score was 0%. This shows that using this criterion possibly reduces the between-study heterogeneity and is possibly the best approach for classification of obesity among children and adolescents. As previously described by Cole TJ et al. (Cole et al., 2005), the BMI-for-age Z score is the best predictor for the adiposity assessment of children on a single occasion (similar to the studies included in our meta-analysis) and not necessarily the best scale for measuring adiposity change overtime. Instead, for predicting the overtime change among the youth, adiposity BMI itself or BMI percentile are better alternatives (Vanderwall et al., 2018).

The possible underlying mechanisms of the shorter LTL with increased adiposity are obtained by performing studies among the adults. The increased markers of oxidative stress, including reactive oxygen substances (ROS), can trigger the negative effects of adiposity on telomere shortening (Bojesen, 2013; Krishna et al., 2015; Yeh and Wang, 2016; Gielen et al., 2018; Salvestrini et al., 2019). Obesity is characterized by high inflammation and oxidative stress (Fernández-Sánchez et al., 2011). Inflammation causes telomere dysfunction in blood *via* increasing the rate of leucocyte turnover, and therefore increasing the rate of replicative senescence. ROS can cause telomere shortening by directly damaging the vulnerable G triplets of the telomeric sequence (Von Zglinicki, 2002). However, regular exercise results in a net decrease in stress hormones, and oxidative stress has been related to increases in telomerase activity in both animals and humans (Simioni et al., 2018; Vicencio et al., 2019). Cortisol also increases ROS production and interferes with antioxidant defenses and increasing oxidative stress in the cell (Espinoza et al., 2017). While the activity of telomerase is generally suppressed in somatic cells, cortisol may inhibit it more and reduce telomere repair (Choi et al., 2008). Therefore, increased oxidative stress and inflammation are all involved in increased telomere abrasion. As revealed by Broer L et al*.* in seven independent cohort studies of more than 11,448 participants, obesity is accompanied with increased leptin concentrations and leptin resistance, and leptin acts as an important pro-inflammatory adipokine and is involved in telomere shortening (Broer et al., 2014). Moreover, fat mass- and obesity-associated genes (FTO) are also another regulator of the telomere length in individuals with obesity; this is done by two direct pathways of Fe(II)- and 2-OG-dependent dioxygenase family and an indirect method *via* the expression of upstream/downstream flanking genes (Zhou et al., 2017). There are multiple possible mechanisms which could affect the cellular mechanisms accountable for telomere attrition and repair, and therefore affect TL (Lyon et al., 2014). However, some of these mechanisms have only been revealed *in vitro*, and it is vague whether they also operate *in vivo* under biologically realistic physiological conditions. A recent study in jackdaws (*Corvus monedula*) found no evidence that oxidative stress shortens telomeres *in vivo* (Boonekamp et al., 2017). A summary of these mechanistic pathways is illustrated in Figure 4.

The article "Leukocyte telomere length and obesity in children and adolescents: A systematic review and meta-analysis" was retracted in 2023. Reason: concerns about the authorship.

**FIGURE 4:** Mechanistic pathways of the possible effects of obesity on leukocyte telomere length shortening among children and adolescents (TL, telomere length; NCD, non-communicable disease).

This study had several limitations. First, the cross-sectional design of the included studies makes it impossible to have a reliable causal inference. Second, due to the limited number of included studies, further prospective studies are warranted to have conclusive results. However, in all the included studies, LTL was assessed with amplifying telomere and single copy gene separately, using a quantitative real-time polymerase chain reaction (RTqPCR). Third, to remove the confounding effects of differences in cell type in telomere length measurement, we measured only LTL, so that the results could be compared with each other; this would minimize the possibility of negative effects of measurement bias on the study results.

## Conclusion

In this systematic review and meta-analysis, for the first time, we identified the shorter LTL among overweight and obese children compared to non-overweight and non-obese ones. Further studies with a longitudinal design are recommended to better elucidate our results. Also, to evaluate adiposity change overtime, more accurate obesity criteria (e.g., BMI or BMI percentile) should be used.

## Data Availability

The original contributions presented in the study are included in the article/Supplementary Material; further inquiries can be directed to the corresponding authors.
